RETRACTED

# Fibrillin-1, induced by Aurora-A but inhibited by BRCA2, promotes ovarian cancer metastasis

**DOI:** 10.18632/oncotarget.3118

**Published:** 2015-02-13

**Authors:** Ziliang Wang, Yang Liu, Lili Lu, Lina Yang, Sheng Yin, Yan Wang, Zihao Qi, Jiao Meng, Rongyu Zang, Gong Yang

**Affiliations:** ^1^ Cancer Institute, Fudan University Shanghai Cancer Center, Shanghai 200032, China; ^2^ Department of Gynecological Oncology, Fudan University Shanghai Cancer Center, Shanghai 200032, China; ^3^ Department of Oncology, Shanghai Medical College, Fudan University, Shanghai 200032, China; ^4^ Department of Biology, Life and Environment Science College, Shanghai Normal University, Shanghai 200023, China; ^5^ Central Laboratory, the Fifth People's Hospital of Shanghai Fudan University, Shanghai 200240, China

**Keywords:** Aurora-A, BRCA2, FBN1, SLUG, Metastasis

## Abstract

While Aurora-A (Aur A) provokes, BRCA2 restrains primary tumorigenesis, the roles of Aur A and BRCA2 in cancer metastasis remains unclear. Here, we show that the metastatic promoting markers SLUG, FBN1, and MMP2, 9, 13 are either stimulated or suppressed by Aur A or BRCA2, but the metastatic suppressors E-cadherin, β-catenin, and p53 are either inhibited or promoted by Aur A or BRCA2, leading to enhanced or reduced cell migration and invasion. Further study suggests that FBN1 inhibits E-cadherin and β-catenin, but stimulates MMP2, 9, 13. Depletion of SLUG abrogates FBN1 and MMP9, but increases E-cadherin, while p53 decreases both SLUG and FBN1. Animal assays demonstrate that FBN1 promotes both ovarian tumorigenesis and metastasis. Clinically, overexpression of BRCA2 or Aur A in ovarian cancer tissues predicts good or poor overall and disease free survivals. High expression of SLUG or FBN1 indicates poor overall survivals, whereas high expression of FBN1 but not of SLUG predicts poor disease free survival. No significant associations between p53 expression and patient survivals were found. Overall, FBN1, acts at the downstream of Aur A and BRCA2, promotes ovarian cancer metastasis through the p53 and SLUG-associated signaling, which may be useful for ovarian cancer diagnosis and treatment.

## INTRODUCTION

Ovarian carcinoma is the leading cause of death in gynecologic cancers due to high metastasis upon being diagnosed, but the detailed mechanism of metastasis remains elusive [1]. The serine/threonine kinase Aurora-A (Aur A), a member of Aurora kinase family reported to induce centrosome amplification, chromosomal instability, and transformation in mammalian cells, is amplified in multiple carcinomas, including ovarian cancer [2, 3]. Breast cancer 2, early onset (BRCA2), as a tumor suppressor functioning in DNA damage repair and genomic stability maintenance, has been linked to several types of cancers [4, 5]. Although we and others have reported that Aur A or BRCA2 promotes or inhibits genomic instability and tumorigenesis through the regulation of cell cycle progression, cytokinesis, and polyploidy [2, 6, 7], the data from literatures indicate that Aur A and BRCA2 may also be involved in cancer metastasis. For instances, the pharmacological or RNA interference-mediated inhibition of Aur A blocked cell migration and adhesion by inhibiting the phosphorylation of the cytoskeletal regulatory protein SRC, whereas the enforced expression of Aur A activated SRC to promote cell migration and adhesion [8]. Moro et al. found that loss of BRCA2 promoted prostated cancer cell invasion through up-regulation of matrix metalloproteinase-9 (MMP9), while downregulation of MMP-9 by inhibition of PI3K/AKT and activation of MAPK/ERKs suppressed cancer cell migration and invasion, limiting the metastatic potential of neoplastic cells [9]. However, the detailed functions of Aur A and BRCA2 in cancer metastasis are unknown.

RETRACTED

Fibrillin-1, namely FBN1, acts as an important and intricate lattice protein in extracellular matrixes to regulate microenvironment [10, 11]. FBN1 binds to each other and forms microfibrils with other proteins, which enables the skin, ligaments, and blood vessels to stretch, and supports more rigid tissues such as nerve, muscle, and lenses of the eyes [12]. Mutations in FBN1 gene can result in Marfan syndrome [13, 14], a disorder that affects the connective tissue supporting the body's joints and organs, and Weill-Marchesani syndrome that causes the eye, heart, and skeletal abnormalities [15]. Growing studies have revealed that FBN1 also functions to regulate organ development and homeostasis [16], integrin α5 assembly [17], and gremlin-1 localization in tumor microenvironment [18]. Guo Q et al. found that the methylation status of the FBN1 promoter was a high specific and sensitive biomarker for colorectal cancer, and the detection of hypermethylated FBNI in stool samples was a useful method for colorectal cancer screening [19]. A recent study revealed that overexpression of FBN1 might indicate ovarian cancer early recurrence and sensitivity to platinum-based chemotherapy [20]. However, the role of FBN1 in ovarian cancer metastasis remains to be uncovered.

The epithelial to mesenchymal transition (EMT) is a molecular event, through which an epithelial cell undergoes transdifferentiation into a mesenchymal phenotype [21]. EMT has been identified to mediate metastasis in various cancers including ovarian cancer. Growing evidence suggests that the EMT transcription factor SLUG (SNAI2) acts to promote cancer cell migration and invasion through suppression of E-cadherin but promotion of MMPs [22]. Haslehurst et al. found that inhibition of SLUG largely reversed the mesenchymal phenotype of ovarian cancer cells, markedly weakened the ability of cell migration and invasion, and resensitized cells to cisplatin treatment [21]. However, the relationship of SLUG and FBN1 has not yet been reported.

RETRACTED

In this study, by silencing or overexpression of Aur A, BRCA2, FBN1, SLUG, or p53 in ovarian cancer cell lines, we investigated the effects of these molecules on ovarian cancer metastasis. We found that FBN1, as a downstream target of Aur A and BRCA2, may promote ovarian cancer metastasis through the p53 and SLUG-associated signaling.

## RESULTS

### Aur A promotes, while BRCA2 inhibits cell migration and invasion

To assess the effect of Aur A or BRCA2 on cell invasion and migration, we delivered Aur A shRNA or BRCA2 cDNA into OVCA429 cells, which generated OVCA429/Aur A shRNA cells and OVCA429/BRCA2 cDNA cells, and Aur A cDNA or BRCA2 shRNA into OVCA420 cells, which generated OVCA420/Aur A cDNA cells and OVCA420/BRCA2 shRNA cells. The immunoblotting analysis showed that the expression level of Aur A was decreased in OVCA429/Aur A shRNA and OVCA420/BRCA2 cDNA cells, but was increased in OVCA420/Aur A cDNA and OVCA420/BRCA2 shRNA cells (Figure 1A). At the same time, the expression level of BRCA2 was increased in OVCA429/Aur A shRNA and OVCA420/BRCA2 cDNA cells, but was decreased in OVCA420/Aur A cDNA and OVCA420/BRCA2 shRNA cells (Figure 1A). These results suggest a mutual suppression between Aur A and BRCR2.

**Figure 1:** The negative correlation between Aur A and BRCA2 regulates the expression levels of metastasis-related proteins **(A)** Detection of Aurora-A or BRCA2 by Western blotting in OVCA429, OVCA429/Aur A shRNA, OVCA429/BRCA2 cDNA, OVCA420, OVCA420/Aur A cDNA, and OVCA420/BRCA2 shRNA cells. **(B)** Immunoblotting analyses of p53, FBN1, and other metastasis-associated proteins. β-actin was used as a loading control.

Next, we detected the expressions of some proteins associated with cell invasion and migration. Silencing of Aur A or overexpression of BRCA2 up-regulated the expressions of p53, E-cadherin and β-catenin, but down-regulated the expressions of MMP2, MMP9, and MMP13 in OVCA429/Aur A shRNA or OVCA429/BRCA2 cDNA cells (Figure 1B), compared with in their control cells. However, overexpression of Aur A or disruption of BRCA2 in OVCA420/Aur A cDNA or OVCA420/BRCA2 shRNA cells resulted in contrary expressions of above proteins, compared with in OVCA429/Aur A shRNA or OVCA429/BRCA2 cDNA cells (Figure 1B).

RETRACTED

We then detected the effects of Aur A or BRCA2 on cell migration and invasion. The results from Figure 2 showed that the number of invaded OVCA429/Aur A shRNA or OVCA429/BRCA2 cDNA cells was much reduced, compared with that of invaded control cells (Figures 2A–2B), but the number of invaded OVCA420/Aur A cDNA or OVCA420/BRCA2 shRNA cells was highly increased, compared with that of their control cells (Figures 2A–2B). We also found by scratch assay that the migration speed of OVCA429/Aur A shRNA or OVCA429/BRCA2 cDNA cells was slowed down after 24 h culture compared with that of control cells (Figures 2C–2D), and that the migration speed of OVCA420/Aur A cDNA or OVCA420/BRCA2 shRNA cells was accelerated after 24 h culture compared with control cells (Figures 2C–2D). These results indicate that Aur A or BRCA2 promotes or inhibits ovarian cancer cell invasion and migration possibly through reducing or inducing p53, E-cadherin, β-catenin expressions, and increasing or decreasing MMP2, MMP9, and MMP13 expressions.

**Figure 2:** Regulation of cell invasion and migration by Aur A or BRCA2 **(A)** Detection of cell migration and invasion by using a high throughput screening multi-well insert 24-well two-chamber plates. **(B)** Quantitative analysis of invaded cells (*P* < 0.05). Error bars = 95% CIs. **(C)** Detection of migration by scratching assay. **(D)** Quantitative analysis of migration speed using migration index (*P* < 0.05). Error bars = 95% CIs.

### FBN1 and SLUG act as down-stream targets of Aur A and BRCA2 to regulate cell migration and invasion

Since FBN1 and SLUG were augmented in OVCA420/Aur A cDNA or OVCA420/BRCA2 shRNA cells, but were decreased in OVCA429/Aur A shRNA or OVCA429/BRCA2 cDNA cells, compared with in control cells (Figure 3A). To examine if FBN1 and SLUG function at the downstream of Aur A and BRCA2 to participate in regulation of cell migration and invasion, we first introduced three siRNAs against FBN1 into OVCA429 cells, and found that the silencing efficiency of FBN1 by siRNA1 was higher than other siRNAs (Figure 3B). Thus, we chose siRNA1 to silence the expression of FBN1 in the following experiments. The results showed that the expression levels of E-cadherin and β-catenin were boosted in OVCA429/FBN1 siRNA, OVCA420/Aur A cDNA/FBN1 siRNA, and OVCA420/BRCA2 shRNA/FBN1 siRNA cells, but the expression levels of MMP2, MMP9, and MMP13 were attenuated, compared with in control cells (Figure 3C). In order to assess whether overexpression of FBN1 directly effects E-cadherin and β-cantenin, we added recombinant FBN1 protein into medium and found that FBN1 suppressed the expressions of E-cadherin and β-cantenin in OVCA420, OVCA429 Aur A shRNA and OVCA420 BRCA2 cDNA cells (Figure 3D). Meanwhile, the migration and invasion of OVCA429/FBN1 siRNA, OVCA420/Aur A/FBN1 siRNA and OVCA420/BRCA2 shRNA/FBN1 siRNA cells were reduced compared with those of control cells (Figures 3E–3F).

RETRACTED

**Figure 3:** Regulation of cell invasion and migration by FBN1 **(A)** Detection of FBN1 and SLUG in OVCA429, OVCA429/Aur A shRNA, OVCA429/BRCA2 cDNA, OVCA420, OVCA420/Aur A cDNA, and OVCA420/BRCA2 shRNA cells. **(B)** Detection of the silencing efficiency of FBN1 in OVCA429 cells with three siRNAs by Western blotting. **(C)** Interruption of FBN1 expression in OVCA429, OVCA420/Aur A and OVCA420/BRCA2 shRNA cells with shRNA altered the expressions of multiple proteins regulated by Aur A and BRCA2. β-actin was used as a loading control. **(D)** Detection of cell migration and invasion by using a high throughput screening multi-well insert 24-well two-chamber plates. **(E)** Detection of migration speed of FBN1-silencing cells by scratch assay. **(F)** Quantitative analysis of migrated and invaded cells (*P* < 0.05). Error bars = 95% CIs.

Next, we introduced three siRNAs against SLUG into OVCA429 cells, and found that siRNA3 was more efficient than other siRNAs in silencing of SLUG (Figure 4A), thus we selected siRNA3 to deplete the expression of SLUG in OVCA429, OVCA420/Aur A cDNA and OVCA420/BRCA2 shRNA cells. The data showed that deprivation of SLUG reduced the expressions of FBN1 and MMP9, but enhanced the expression of E-cadherin in resulting cells, compared with in their control cells (Figure 4B). These data suggest that FBN1 may function as a downstream target of SLUG to regulate cell migration and invasion.

**Figure 4:** Upregulation of FBN1 by SLUG and effects of FBN1 on tumorigenesis **(A)** Knockdown of SLUG with three siRNA detected by Western blotting in OVCA429. **(B)** Knockdown of SLUG with SiRNA detected by Western blotting in OVCA429, OVCA420/Aur A cDNA and OVCA420/BRCA2 shRNA cells and immunoblotting analysis of metastasis-associated proteins. **(C)** Detection of p53, SLUG and FBN1 in SKOV3 cells induced by p53 cDNA. **(D–F)** *In vivo* tumorigenesis examined by animal assays. **(G)** Dissection of xenograft tumors. **(H)** Quantitative analyses of the numbers of the nodules formed in animals (*P* < 0.025 or *P* < 0.05). Error bars = 95% CIs. **(I)** Quantitative analyses of the weights of the nodules dissected from mice (*P* < 0.025 or *P* < 0.05). Error bars = 95% CIs. β-actin was used as the loading control.

It is well-known that p53 suppresses cell migration and invasion that is associated with Aur A and BRCA2 [26, 27], so we wondered whether the altered expressions of SLUG and FBN1 were linked with p53 expression levels in ovarian cancer cells. To address this issue, we introduced a wild type p53 cDNA into p53 null SKOV3 cells and found that overexpression of p53 inhibited the expressions of SLUG and FBN1 (Figure 4C). To further confirm this notion, we treated low Aur A but high BRCA2 expressing cells with p53 shRNA, and low BRCA2 but high Aur A expressing cells with p53 cDNA. The results showed that overexpression of p53 suppressed the expressions of SLUG and FBN1 in OVCA429/p53 cDNA, OVCA420 Aur A cDNA/p53 cDNA, or OVCA420 BRCA2 shRNA/p53 cDNA cells (Figures 4D–4E), and that silencing of p53 enhanced the expressions of SLUG and FBN1 in OVCA420/p53 shRNA, OVCA429 Aur A shRNA/p53 shRNA, or OVCA429 BRCA2 cDNA/p53 shRNA cells (Figures 4D–4E). Thus, we conclude that Aur A amplification or BRCA2 deficiency promotes ovarian cancer cell migration and invasion through suppression of p53, but induction of SLUG/FBN1.

RETRACTED

### FBN1 promotes ovarian cancer tumorigenesis and metastasis

To further explore the association of FBN1 with tumorigenesis, we performed animal assays with cells expressing FBN1 shRNA or scrambled shRNA (control). Tumor sizes were measured every 7 days. OVCA429/control cells generated the mean tumor volume of 497.3 mm^3^, while OVCA429/FBN1 shRNA cells generated a reduced tumor volume of 234.6 mm^3^ at 42 days (Figure 4F, *p* < 0.05). Tumor sizes formed by OVCA420/Aur A cDNA/FBN1 shRNA and OVCA420/Aur A cDNA/control cells at 42 days were 198.4 mm^3^ and 345.9 mm^3^, respectively (Figure 4G, *p* < 0.05). The tumor volume formed by OVCA420/BRCA2 shRNA/FBN1 shRNA cells was lowered to 144.8 mm3 compared with the tumor size of 346.3 mm^3^ formed by OVCA420/BRCA2 shRNA cells at 42 days (Figure 4H, *p* < 0.05). In addition, the mean numbers of tumor nodules in peritoneal cavity of each animal injected with OVCA429/FBN1 shRNA, OVCA420/Aur A cDNA/FBN1 shRNA, and OVCA420 BRCA2 shRNA/FBN1 shRNA cells were 7, 0, and 0, respectively, while those of tumor nodules generated by their control cells were 81, 6, and 6, respectively (Figure 4I–4J). The mean weights of tumor nodules per mouse injected with FBN1 shRNA expressing cells were 0.226, 0, and 0 grams, respectively, but those of control tumor nodules were 6.54, 0.297, and 0.263 grams, respectively (Figure 4K). These data suggest that FBN1 promotes both ovarian tumorigenesis and metastasis.

### Clinical correlations with expressions of BRCA2, Aur A, SLUG, FBN1, and p53

To investigate whether expressions of Aur A, BRCA2, SLUG, FBN1, and p53 were associated with clinical pathological characteristics of ovarian cancer patients, we performed immunostaining using antibodies to BRCA2, Aurora-A, SLUG, FBN1 or p53 in a tumor tissue microarray consisting of 150 high-grade ovarian serous carcinomas and 30 normal ovarian tissues. We first analyzed the associations between the expressions of Aur A, BRCA2, p53, SLUG and FBN1 and the patients’ characteristics, and found that no statistical significance was found between the expressions of these proteins and age or ascites. The expressions of BRCA2 and FBN1, but not of Aur A, SLUG and p53, were significantly associated with FIGO stage (*P* < 0.05). With regard to chemoresponse, only did BRCA2 reach the statistical significance (Table 1). No expression of Aur A, SLUG, FBN1, or p53, but not of BRCA2 was detected in normal tissues (data not shown).

RETRACTED

**Table 1:** Association of Aurora A, BRCA2, FBN1 and SLUG expressions with patient clinical characteristics

	Aurora A			BRCA2			FBN1			SLUG		
	H	L	*P*	H	L	*P*	H	L	*P*	H	L	*P*
**Age at diagnosis (y)**												
≤57	35	46		13	68		43	38		41	40	
> 57	31	38		13	56		43	26		35	34	
Total	66	84	0.481	26	124	0.406	86	64	0.165	76	74	0.560
**FIGO stage**												
IIIc	62	72		20	114		81	53		70	64	
IV	4	12		6	10		5	11		6	10	
Total	66	84	0.086	26	124	0.036*	86	64	0.025*	76	74	0.198
**Ascites(ml)**												
≤ 1500	38	50		13	75		54	34		43	45	
> 1500	28	34		13	49		32	30		33	29	
Total	66	84	0.470	26	124	0.220	86	64	0.154	76	74	0.359
**Chemoresponse**												
Chemoresistant	32	33		5	60		37	28		36	29	
Chemosensitive	33	52		22	63		48	37		41	44	
Total	65	85	0.128	27	123	0.002*	85	65	0.535	77	73	0.246

H, High expression

L, Low expression

* Statistical significance (*P* < 0.05)

We further found that the nuclear score for BRCA2 was negatively correlated with Aurora-A, FBN1, SLUG or p53 staining in tumor tissues (*P* < 0.05), as evidenced by the representative images showing that high expression of BRCA2 corresponded to low expressions of Aur A, FBN1, SLUG or p53 in the same tissues (Figure 5A), or vice versa (Figure 5B). The expressions between two of Aur A, FBN1, SLUG and p53 were positively correlated (*P* < 0.05). The nuclear accumulation of BRCA2 was significantly associated with good overall survival (24 of 148 patients, or 16.2%; *P* = 0.015) and disease-free survival (24 of 143 patients, or 16.8%; *P* = 0.021; Figure 5C). Strong staining for Aurora-A was significantly associated with poor overall survival (64 of 148 patients, or 43.2%; *P* = 0.027) and disease-free survival (62 of 143 patients, or 43.4%; *P* = 0.033; Figure 5D). The staining of SLUG was significantly associated with poor overall survival (75 of 148 patients, or 50.7%; *P* = 0.018), but not with disease-free survival (73 of 143 patients, or 51%; *P* = 0.076; Figure 5E). The strong staining of FBN1was significantly associated with poor overall survival (86 of 148 patients, or 58.1%; *P* = 0.025) and disease-free survival (82 of 143 patients, or 57.3%; *P* = 0.034; Figure 5F). Statistically, patients with high expression of BRCA2 (mean, 38.2 months), or low expressions of Aur A (mean, 43.4 months), SLUG (mean, 41.2 months), or FBN1 (mean, 46.2 months) lived longer than patients with low expression of BRCA2 (mean, 27.4 months; *P* < 0.05), or high expressions of Aur A (mean, 29.4 months; *P* < 0.05), SLUG (mean, 34.0 months; *P* < 0.05), or FBN1 (mean, 30.1 months; *P* < 0.05) (Supplementary Table 1). In term of disease-free survival, patients with low expression of BRCA2 (mean, 17.9 months) or high expressions of Aur A (mean, 13.6 months), SLUG (mean, 15.8 months), or FBN1 (mean, 14.5 months) relapsed earlier in the course of the disease than did patients with high expression of BRCA2 (mean, 13.5 months; *P* < 0.05) or low expressions of Aur A (mean, 20.8 months; *P* < 0.05), SLUG (mean, 21.0 months; *P* < 0.05), FBN1 (mean, 21.0 months; *P* < 0.05) (Supplementary Table 2). However, the staining of p53 was not significantly associated with poor overall survival (73 of 143 patients, or 51.0%; *P* = 0.078) and disease-free survival (86 of 148 patients, or 58.1%; *P* = 0.127; Figure 5G).

RETRACTED

**Figure 5:** Immunohistochemical analyses of Aur A, BRCA2, FBN1 and SLUG expression and correlation in high-grade ovarian serous carcinoma and the associations of the molecules with patient survivals Representative images from tissue microarray stained for BRCA2 and Aur A. **(A)** high expression of BRCA2 in nuclei is correlated with low expression of Aur A, FBN1 and SLUG in the same core of high-grade ovarian carcinoma (× 400). **(B)** high expressions of Aur A, FBN1 and SLUG expression are correlated with low nuclear accumulation of BRCA2 in the same core of high-grade ovarian carcinoma (× 400). **(C)** the favorable overall and disease-free survivals (*P* = 0.015, *P* = 0.021) are associated with the accumulated nuclear staining of BRCA2. **(D)** the poor overall and disease-free survivals (*P* = 0.027, *P* = 0.033) are associated with strong staining of Aur A. **(E)** the poor overall survival (*P* = 0.018) but not the disease-free survival (*P* = 0.076) is associated with the strong expression of SLUG. **(F)** the poor overall survival (*P* = 0.025) but not the disease-free survival (*P* = 0.779) is associated with the strong expression of FBN1. H, high expression; L, low expression.

In univariate Cox regression analysis (Supplementary Table 3), we found that residual tumors, resistant sensitivity, Aur A, BRCA2, and FBN1 were significantly associated with DFS outcome, and that ascites, FIGO, Aur A, BRCA2, SLUG, and FBN1 were significantly associated with OS outcome. In multivariate Cox regression analysis, ascites, FIGO, FBN1, and SLUG were significantly associated with OS outcome (Supplementary Table 4), and residual tumors, resistant sensitivity, SLUG were significantly associated with DFS outcome (Supplementary Table 5). These data suggest that the expression of Aurora-A, FBN1, SLUG or BRCA2 can independently predict the outcomes of patients with high-grade serous ovarian cancer.

RETRACTED

We also analyzed the associations of the expression ratios between Aurora-A, FBN1 or SLUG and BRCA2 with progression in high-grade serous ovarian carcinomas. As shown in Figure 6, the increased ratios of Aur A (simplified as A), SLUG (simplified as S) or FBN1 (simplified as F) to BRCA2 (simplified as B) (Ap/Bn, Sp/Bn, Fp/Bn; p for positive, n for negative) predicted poor overall survival (*P_A/B_* = 0.002, *P_S/B_* = 0.003 and *P_F/B_* = 0.001) (Figures 6A–6C) and disease-free survival (*P_A/B_* = 0.01, *P_S/B_* = 0.02 and *P_F/B_* = 0.027) (Figures 6A–6C), compared with the low ratios of Aur A, FBN1, or SLUG to BRCA2 (An/Bp, Sn/Bp or Sn/Bp). No statistical significance was found between other ratios in terms of overall and disease-free survivals (data not shown).

**Figure 6:** Association of the expression ratios between Aurora-A, SLUG, or FBN1 and BRCA2 with patient survivals **(A–C)** The increased ratios of Aurora-A, SLUG or FBN1 to BRCA2 (Ap/Bn, Sp/Bn, or Fp/Bn) are associated with poor overall survival (*P_A_* = 0.002, *P_F_* = 0.003 or *Ps* = 0.001) and disease-free survival (*P_A_* = 0.010, *P_F_* = 0.020 or *Ps* = 0.027), compared with the decreased ratios of Aurora-A, SLUG or FBN1 to BRCA2 (An/Bp, Sn/Bp, or Fn/Bp).

## DISCUSSION

In this study, we demonstrate that activation of Aur A or inactivation of BRCA2 stimulates ovarian cancer cell migration and invasion through upregulation of FBN1, SLUG, MMP2, MMP9, MMP13, but downregulation of p53, E-cadherin, and β-catenin. Knockdown of FBN1 inhibits cell migration and invasion, while silencing of SLUG decreases the FBN1 expression. The tumor suppressor p53, suppressed by Aur A but promoted by BRCA2, diminishes SLUG and FBN1 expressions, indicating that p53 negatively regulates SLUG and FBN1. Clinically, we show that high expressions of Aur A, FBN1 or SLUG, and low-expression of BRCA2 were significantly associated with poor disease-free and/or overall survivals, but high expression of p53 was not associated with patient survivals although p53 is commonly mutated and highly expressed in high grade serous ovarian cancer tissues, which is consistent with a previous study [28].

RETRACTED

Recently, increasing studies have shown that activation of Aur A or inactivation/mutation of BRCA2 is associated with cancer metastasis [29–33]. In spite that different signal pathways have been reported, the tumor suppressor p53 may still play an important role in terms of the Aur A and BRCA2 status during cancer metastasis. Studies have shown that Aur A phosphorylates p53 to abrogate its transactivation function and stabilization in cancer cells [34, 35]. Although p53 is reported to repress BRCA2 expression [36] and BRCA2 interacts with p53 to maintain genomic integrity [37], the interactive relationship between p53 and BRCA2 is not clear. Thus, how Aur A and BRCA2 regulate the expression of p53 is intricate in ovarian cancer cells. Since p53 and SLUG are dominantly reported to be mutually suppressed in cancer cells [38–40], our finding that p53 inhibits the SLUG-mediated FBN1 expression may be rational. However, because p53 is commonly mutated in high-grade serous ovarian cancer, how the signal pathway is regulated by Aur A and BRCA2 still needs further study.

Although the mutation of FBN1 is a main pathogenesis of Marfan syndrome and Weill-Marchesani syndrome [41, 42], the overexpression of FBN1 is also detected in cancer tissues [43]. Several studies have shown that FBN1 is associated with TGF-beta signaling [44, 45], while the TGF-beta signaling is reportedly to induce EMT that may in turn regulate the expressions of E-cadherin, beta-catenin, and MMPs [46–49]. Thus, FBN1 may indirectly suppress the expressions of E-cadherin, beta-catenin, and induce the expressions of MMPs through the TGF-beta-mediated signaling, although it is possible that FBN1 may function as a secretive matrix protein to interact with membrane receptors, which thereby activates additional signal pathways to regulate EMT and the expressions of these proteins in ovarian cancer cells. However, more investigations are definitely needed to validate these hypotheses.

Taken together, we have uncovered a mechanism in human ovarian cancer that FBN1, stimulated by Aur A but inhibited by BRCA2, promotes ovarian cancer metastasis possibly through the p53 and SLUG-associated signaling (Figure 7), which may provide some novel insights to improve ovarian cancer diagnosis and treatment.

**Figure 7:** A schematic diagram of how Aur A and BRCA2 regulate ovarian cancer metastasis through p53/SLUG-mediated FBN1 signalling The expression of p53, suppressed by Aur A, but promoted by BRCA2, inhibits the expressions of SLUG and FBN1, which accentuates the expressions of E-cadherin and β-catenin, but attenuates the levels of MMP2, MMP9 and MMP13 to eventually abrogate the ovarian cancer metastasis.

RETRACTED

## MATERIALS AND METHODS

### Cell lines and cell culture

Human ovarian epithelial cancer cell lines SKOV3 with p53 null, OVCA420 with low Aur A and high BRCA2, and OVCA429 with low BRCA2 and high Aur A, and retroviral packaging cells (Phoenix amphotropic cells) were as gifts from Dr. Yinghua Yu’ lab (Obstetrics and Gynecology Hospital of Fudan University, Shanghai, China), or purchased from American Type Culture Collection (ATCC, USA). SKOV3, OVCA420 and OVCA429 cells were maintained in Roswell Park Memorial Institute (RPMI) 1640 medium, phoenix cells were cultured with Deulbecco's Modified Eagle Medium (DMEN). Both media were supplemented with 10% fetal bovine serum, 2 mM l-glutamine, penicillin (100 units/ml), and streptomycin (100 μg/ml). Cells were incubated at 37°C in an atmosphere of 5% CO2 and 95% air.

### Plasmids construction, cell transfection and viral infection

To enhance the expression of Aur A and BRCA2, human wild type cDNAs of Aur A and BRCA2 were inserted into pBabe/puromycin or pCIN-neomycin, respectively. Viruses produced from phoenix cells transfected with pBabe/Aur A were collected to infect OVCA420 cells and to establish the Aur A overexpression cell line OVCA420/Aur A using the previously published methods [5, 23]. The control cell line was generated by infection with viruses containing empty vector. pCIN/BRCA2 cDNA was transfected into OVCA429 by using Fugene 6 (Roche) according to manufacturer's instruction, to generate the BRCA2 overexpression cell line OVCA429/BRCA2. Cells transfected with pCIN were used as controls. The resulting cells were selected with puromycin (1.5–2.0 μg/ml) or neomycin (0.5–2.5 mg/ml) for 7–14 days.

To silence the expression of Aurora-A and BRCA2, the DNA oligonucleotides used to generate shRNAs against the open reading frame of mRNA were 5′-GUCUUGUGUCCUUCAAAUU-3′ (Aurora-A shRNA) and 5′-ACAAUUACGAACCAAACCG-3′ (BRCA2 shRNA). pBabe/U6-puromycin-Aur A shRNA and pBabe/U6-neomycin-BRCA2 shRNA were generated according to the previously reported method [5]. The control vector was similarly constructed by directly inserting a scrambled shRNA (Control shRNA) into pBabe/U6-neomycin. Retroviral particles were generated by using the same method mentioned above, and were used to infect and generate new cell lines including OVCA429/Aur A shRNA and OVCA420/BRCA2 shRNA. Corresponding control cell lines were made by infection of viruses expressing the scrambled shRNA (control shRNA). The infected cells were selected with puromycin (1.5–2.0 μg/ml) or neomycin (0.5–2.5 mg/ml) for 7–14 days.

To overexpress p53 in SKOV3 cells, human wild type p53 cDNA was inserted into pBabe/puromycin vector. Viruses generated from phoenix cells transfected with pBabe/p53 were used to establish the p53 overexpression cell line SKOV3/p53 using the same method described above [5, 23]. The resulting cells were selected with puromycin (1.5–2.0 μg/ml) for 7–14 days.

RETRACTED

### RNA interference with FBN1 and SLUG siRNA

Three small interfering RNAs (siRNAs) targeting FBN1 (siRNA1: sense : 5′GGGAGGAAAUUGCAUU AAUTT 3′, antisense: 5′AUUAAUGCAAUUUCCUCCCTT 3′; siRNA2: sense: 5′GGCGAUGUGAGAUCAACAUTT 3′, antisense:5′AUGUUGAUCUCACAUCGCCTT 3′; siRNA3: sense : 5′CGUGGCUUCAUUCCAAAUATT 3′, antisense: 5′UAUUUGGAAUGAAGCCACGTT 3′), or SLUG (siRNA1: sense : 5′GACCCACACAUUACCUUGUTT 3′, antisense: 5′ACAAGGUAAUGUGUGGGUCTT 3′; siRNA2: sense: 5′GCACAAACAUGAGGAAUCUTT 3′, antisense: 5′AGAUUCCUCAUGUUUGUGCTT 3′; siRNA3: sense : 5′GCAGACCCAUUCUGAUGUATT 3′, antisense: 5′UACAUCAGAAUGGGUCUGCTT 3′) gene were purchased from GenePharma (Shanghai, China). These ds-siRNAs were respectively transfected into OVCA429, OVCA420/Aur A and OVCA420/BRCA2 shRNA cells with Lipofectamine. Scrambled siRNAs were designed by company and used for siRNA controls.

### Cell invasion and migration

To test cell invasion, we used a high throughput screening multi-well insert 24-well two-chamber plate (BD Biosciences, San Jose, CA), with an 8-μm (pore size) polycarbonate filter between chambers. 3 × 10^4^ cells were added in upper chamber and allowed to invade at 37°C for 24 hours toward a lower reservoir containing medium plus fibronectin (20 μg/mL). The cells were then fixed in 100% methanol for 30 minutes and stained with Giemsa solution for 10 minutes. The invasive cells were counted as those passed through the membrane separating the chamber. All cells were counted at × 200 magnification under a microscope. The assay was repeated three times with duplicate.

To examine cell migration, cells were incubated in 6-well plate overnight to yield monolayer confluence for scratch assay. Scratches were made using a pipette tip and photographed immediately (time 0) and 24 hours’ later. The distance migrated by the cell monolayer to close the scratch area during the time period was measured. Results were analyzed as migration index, which was the ratio of the cell migration distance at 24 h to that at 0 h. The assay was carried out in triplicate and repeated three times.

### Cell treatment and immunoblotting analysis

The recombinant FBN1 protein (rFBN1), purchased from Abova (Taiwan) corporation, was prepared at the stock concentration of 0.08 μg/μl and the working concentration of 20ng/ml. Cells were collected and subjected to Western blot analysis after treatment with rFBN1 for 24 hours. To analyze protein expressions by Western blot, we prepared cell lysates at 75% of confluence using 500 μL of radioimmunoprecipitation assay buffer (RIPA, 25 mM Tris–HCl at pH 7.6, 150 mM NaCl, 1% Nonidet P-40, 1% sodium deoxycholate, and 0.1% sodium dodecyl sulfate). The protein concentration of each lysate was determined with a Bio-Rad protein assay kit (Hercules, CA). Immunoblotting analyses were performed as described previously [2, 24]. Antibodies against the following proteins were obtained from Santa Cruz Biotechnology: BRCA2, FBN1, SLUG, MMP2, MMP9, MMP13, p53, and E-cadherin. Antibodies against the following proteins were from Cell Signaling Technology (Danvers, MA): Aur A, β-catenin, and β-actin. The secondary antibodies were F(ab)2 fragments of donkey anti-mouse immunoglobulin (product NA931) or of donkey anti-rabbit immunoglobulin (product NA9340) linked to horseradish peroxidase from Amersham Biosciences (Little Chalfont, Buckinghamshire, UK). Immunoblotting reagents were from an electrochemiluminescence kit (Amersham Biosciences).

RETRACTED

### Animal assays

OVCA429, OVCA420/Aur A, and OVCA420/BRCA2 shRNA cells stably transfected with FBN1 shRNA or scrambled shRNA by retroviral infection were used for animal assay. To generate tumor growth *in vivo*, 1 × 10^7^ cells of each cell line were subcutaneously injected into 4- to 6-week-old BALB/c athymic nude mice (Department of Laboratory Animal, Fudan University). The animal experiments were approved by the Institutional Animal Care and Use Committee of Fudan University and performed following Institutional Guidelines and Protocols. Each cell line was bilaterally injected into eight mice, for a total of 16 injections. The longest diameter “a” and the shortest diameter “b” of tumors were measured and the tumor volume was calculated with the use of the following formula: tumor volume (in mm^3^) = a × b^2^ × 0.52 [2], where 0.52 is a constant to calculate the volume of an ellipsoid. When a tumor reached 1.0 cm in diameter, the mouse was sacrificed and the tumors were weighed. Four tumors per cell line were excised, fixed in 10% formalin overnight, and subjected to routine histological examination by investigators who were blinded to the tumor status. For the intraperitoneal injection group, six mice were used for each cell line and each mouse received one injection of 2 × 10^7^ cells. Mice were observed for lethargy, poor appetite, and abdominal enlargement, and sacrificed timely before natural death occurred. Tumor nodules and ascites were counted, weighed, or measured for their numbers, weights, and volumes. Animal assays were repeated twice.

### Patient information

Ovarian tissue samples from patients with primary high grade epithelial ovarian cancer or fallopian tube diseases (for collection of normal ovarian tissues), who had undergone initial surgery at Fudan University Shanghai Cancer Center between June 2005 and December 2010, were included in this study. 150 correlative patients were identified with the updated follow-up information until January 6th, 2014. Histopathologic diagnoses were based on WHO criteria; tumor grade based on Gynecologic Oncology Group criteria; each case was assigned as an information consent form and was approved by Ethics Committee of Fudan University Shanghai Cancer Center. The management of relapsed disease was stratified based upon the amount of time that has elapsed between the completion of platinum-based treatment and the detection of relapse, known as the platinum-free interval (PFI). Patients with a PFI of six months or longer were considered to have “platinum sensitive” disease. Patients with a PFI of less than six months were considered to have “platinum-resistant” disease. The mean age of the 150 patients was 57 years (ranging from 31 to 85 years) (Table 1). With regard to surgical disease stage, 134 patients (89.3%) had stage IIIc disease, and 16 (10.7%) had stage IV disease. The mean ascites was 1500ml (ranging from 0 to 10000ml). The mean follow-up interval was 33 months (ranging from 9 to 131 months). Until the last follow-up, 46 patients (30.7%) were alive, 102 (68%) were dead, and 2 (1.3%) lost the follow-up. The overall survival rate at 3 years was 48.7%, 84 patients (56.8%) had “platinum sensitive” disease and 64 patients (43.2%) had “platinum-resistant” disease.

RETRACTED

### Immunohistochemical staining

A tissue microarray consisting of core samples from 30 normal human ovarian tissues and 150 human ovarian carcinomas described above. The TMA was made technically according to the previously published method [6]. The expressions of Aur A, BRCA2, FBN1, SLUG, and p53 were detected by immunohistochemical staining. Antibodies used to detect Aur A, BRCA2, FBN1, SLUG, and p53 were described as above. The paraffin-embedded sections were pre-treated and stained with antibodies by using the previously reported method [6, 25]. The secondary antibodies against mouse or rabbit IgG were supplied in an IHC kit (#CW2069) from Beijing CoWin Bioscience Co. Ltd (Beijing, China). Results were separately judged, evaluated, and scored by two pathologists (Drs. Bin Chang and Xiaoyu Tu) without knowing the patients’ information. The expressions of Aur A, BRCA2, SLUG and FBN1 were determined based on the percentage of positive cancer cells and the staining intensity. The percentage of positive cells (PPC) was divided into five levels as follows: 0 =< 5% of positive cells, 1 = 5~25%, 2 = 25~50%, 3 = 50~75%, and 4 => 75% of positive cells. The intensity of staining (IS) was classified as 0 = no staining, 1 = weak staining (light yellow), 2 = moderate staining (yellow brown), and 3 = strong (dark brown). As for the negative control, the primary antibody was replaced with PBS. The score of the protein expressions was determined by PPC × IS, which was divided as 0~4 for weak staining, 4~8 for intermediate staining, and 8~12 for strong staining. For clinical association analysis, the final score was graded as “low” for < 4 and “high” for ≥ 4.

RETRACTED

### Statistical analysis

All *in vtiro* data were analyzed by the Student *t* test. Tumor growth, and statistical significance between the protein expressions and the patient information including age, FIGO stages, ascites, and chemoresponse was analyzed by Chi-square test, while the overall and disease free survivals were statistically analyzed by using SPSS software (version 18.0). *P* < 0.05 was considered statistically significant.

## SUPPLEMENTARY TABLES


